The article "Music Emotion Analysis Based on PSO-BP Neural Network and Big Data Analysis" was retracted in 2023. Reasons: unreliable results or conclusions; concerns about the data; concerns about the peer review; concerns about the citations.

# Music Emotion Analysis Based on PSO-BP Neural Network and Big Data Analysis

**DOI:** 10.1155/2021/6592938

**Published:** 2021-09-03

**Authors:** Chen Xi

**Affiliations:** School of Music, Shaanxi Normal University, Xi'an, Shaanxi 710119, China

## Abstract

The current music teaching can effectively improve students' music emotional expression indirectly. How to use the PSO-BP neural network to realize the quantitative research of music emotional expression is the current development trend. Based on this, this paper studies the influence factors of music emotion expression based on PSO-BP neural network and big data analysis. Firstly, a music emotion expression analysis model based on PSO-BP neural network algorithm is proposed. The autocorrelation function is used to simulate the emotion expression information in music. Through the maximum value of the autocorrelation function curve in the detection process, the vocal music signal is restored, and then the emotion expressed is analyzed. Secondly, the influence factors of PSO-BP neural network algorithm in music emotion expression are analyzed. The improved PSO-BP neural network algorithm and multidimensional data model are used for comprehensive analysis to accurately analyze the emotion in music expression, and the fuzzy evaluation method and analytic hierarchy process are used for quality evaluation. Finally, the validity of the music emotion analysis model is verified by many experiments.

## 1. Introduction

The related research of music emotion expression started earlier and involved a wide range of content [1]. In addition, in the process of studying the influence of intelligent algorithm on music emotion expression, PSO-BP neural network is also a hot spot. From the analysis of the influence of music on emotion, in addition to the improvement of students' music literacy [2]. It also involves psychological adjustment, which has been widely concerned by the industry since the 1930s [3]. In the research theory, the evaluation of music simulation is considered to be the most important part, hoping to improve the efficiency of music emotional expression in this way [4]. The institute of music emotion expression has also carried out relevant research, and various simulation models emerge in endlessly, such as analytic hierarchy process, factor judgment method, hierarchical expression method, and so on [5]. At present, the research on the influencing factors of music emotion expression in the industry has the problem of low intelligence level, and many experts and scholars have studied music emotion analysis [6]. Sakaki et al. have improved the emotional representation method of music in the process of expression according to the different types of audio signals in different environments [7]. Hirschfeld et al. conduct a differentiated analysis based on the expression process of music emotions and realize specific representations of music emotion characteristics according to fixed key information [8]. Peng et al. use the normalization method to collect the data signal input to the model and realize the information simulation processing of the data signal through the PSO-BP neural network algorithm [9]. Sanglerdsinlapachai et al. summarize the current music sentiment analysis methods, classify them according to their recognition principles, and conduct a differentiated analysis of the advantages and disadvantages of different types of music sentiment analysis process [10]. According to different types of music data information, Carvalho and Plastino have performed ultra-high discrimination recognition of existing music sentiment analysis methods and realized high-accuracy analysis in terms of their composition and expression methods [11]. Based on the existing 5G technology, Huang et al. perform multidimensional quantification of different types of music sentiment analysis processes and realize the construction of regular functions according to their differences [12]. In response to the high error rate in the process of music sentiment analysis, Sze et al. proposed a hyperquantitative music sentiment analysis method in combination with audio dedusting methods [13]. Samek et al. have verified the effectiveness of the music emotion evaluation system in the PSO-BP neural network through practice, and the results show that the innovative PSO-BP neural network analysis method can effectively perform high accuracy on different types of databases [14]. In summary, it can be seen that, in the current research of music emotion expression, most of the music emotion analysis methods have not constructed a music emotion expression influence evaluation model based on the improved PSO-BP neural network algorithm [15].

In the research of processing signals and performing sentiment analysis, scholars have confirmed that the neural network algorithms can efficiently and accurately complete the feature extraction and internal correlation analysis of data information and has formed a neural network algorithm [16–19]. It is the core data analysis system and evaluation standard, but there are few breakthroughs and advances in the analysis of emotional uniqueness of music signals and the adaptive discrimination of emotional types [20, 21]. Therefore, although research scholars have done a lot of basic research on the expression of music emotion, the research results are relatively few [22].

Under this background, this paper puts forward the influence analysis model of music emotion based on improved PSO-BP neural network algorithm. Compared with the existing research results, the innovation of this paper is to propose a PSO-BP neural network simulation system based on the improved PSO-BP neural network algorithm. On this basis, the system cannot only realize the daily recording and storage of the information data contained in the process of music expression under different PSO-BP neural networks, but can also make full use of the difference of timbre and frequency in the process of music emotion expression and realize the closed-loop evaluation of music emotion expression in the process of PSO-BP neural network through data comparative analysis. This paper studies the music emotion evaluation model based on PSO-BP neural network algorithm; the rest of this paper is mainly divided into four sections. In Section 2, we discuss the application of PSO-BP neural network algorithm and big data system in music emotion analysis model. In Section 3, we study music emotion analysis model based on PSO-BP neural network algorithm and big data analysis. In Section 4, we analyze and discuss the experimental results. In Section 5, the conclusion and limitation of this paper are performed.

## 2. The Application of PSO-BP Neural Network Algorithm and Big Data System in Music Emotion Analysis Model

In the process of finding the optimal solution, the commonly used algorithms are PSO-BP neural network algorithm, mountain climbing algorithm, simulated annealing algorithm, and PSO-BP neural network algorithm [23]. PSO-BP neural network algorithm, like simulated annealing algorithm, is a general optimization algorithm [24]. At present, it has been well applied in many engineering fields, such as production scheduling, control engineering, computer vision, PSO-BP neural network, image processing, and accurate query of database information [25]. At present, most of the database applications are in the computer teaching industry, mainly for the automatic classification of data. Most of the classification systems with the best application effect are based on BP neural network algorithm [26]. In addition, in the signal processing of music data, different types of optimization methods have emerged, especially in the process of music sentiment analysis. PSO-BP neural network algorithm is an optimization improvement based on PSO-BP neural network algorithm and has been comprehensively developed in recent years, and optimization methods in time domain and frequency domain are also emerging [27]. Among many methods for quantitative analysis of music emotion expression results, PSO-BP neural network algorithm has been paid attention to in recent years. In the process of audio signal analysis and processing, the mathematical modeling by PSO-BP neural network algorithm is to determine the mathematical relationship between many factors of gray system. In the process of music emotion analysis, it is through the feature extraction of audio signal, according to the extraction results, to complete the distinction of different signals in terms of emotional differences. Compared with the conventional music emotion analysis method, this signal processing method has higher accuracy and reliability. In the process of emotional analysis of music, common reference indicators are shown in Table 1.

## 3. Music Emotion Analysis Model Based on PSO-BP Neural Network Algorithm and Big Data Analysis

### 3.1. Construction Process of Music Emotion Analysis Model Based on PSO-BP Neural Network

The music signal processing process of PSO-BP neural network algorithm is shown in Figure 1. With the deepening research of PSO-BP neural network algorithm in audio signal processing by scholars, in the aspect of theoretical research, the English version of international academic journals founded by the UK published many researches on this theory, especially in the application of music system. These can be analyzed and processed by using PSO-BP neural network algorithm theory. In addition, we need to obtain the key features of the signal through the neuron node.

The PSO-BP neural network algorithm is a backpropagation neural network algorithm optimized with the characteristics of particle swarms. The algorithm combines the BP drop to adjust the weights, through the revised analysis of the network weights and thresholds according to the idea of particle swarm optimization, data training, and deep learning in the BP neural network. This is because the particle swarm can roughly search the data on a global scale to obtain an initial solution, which reduces the difficulty of analyzing the BP neural network, thereby improving the efficiency and accuracy of data analysis (rate).

The first step is to measure the degree of association according to the relationship or similarity between the factors in the neuron nodes. The basic idea is to rank according to the degree of association. In the application, the original data matrix is initialized, and then the reference data column is established. The music signal *w*_*t*_^(0)^(*x*) can be marked as follows:

(1) $$\begin{array}{c} w_{t}^{\left(0\right)}\left(x\right)=\sqrt{\frac{w_{1}^{\left(0\right)}\left(x\right)+w_{2}^{\left(0\right)}\left(x\right)+\cdots +w_{n}^{\left(0\right)}\left(x\right)}{n},} \end{array}$$

where *x* is the signal factor and *n* is the dimension of the signal.

The second step is to calculate the absolute difference between the subfactor and the main factor at a certain time.

(2) $$\begin{array}{c} \Delta_{t}\left(i,x\right)=iw_{t}^{\left(i\right)}\left(x\right)-lw_{t}^{\left(l\right)}\left(x\right), \end{array}$$

where *i* is the neural layer, *l* is the reference data column, and *t* is the individual in different data columns.

The third step is to calculate the correlation degree *ζ*_*i*_(*x*) between subfactors and main factors; the equation is as follows:

(3) $$\begin{array}{c} {\left|\zeta_{i}\left(x\right)\right|}^{2}=\frac{\zeta \sqrt{l^{2}+t^{2}}}{\sqrt{n}}{\left|w_{t}^{\left(l\right)}\left(i\right)-w_{t}^{\left(l\right)}\left(x\right)\right|}^{2}, \end{array}$$

where *ζ* is the resolution coefficient.

Therefore, according to the mark of the music signal in the above equation, the absolute difference calculation and the correlation degree calculation of the marked music signal at different times can be calculated according to the inherent relationship between the absolute difference and the correlation degree. Realize the disturbance analysis and calculation of different factors. This is because in the process of processing data, through the quantitative analysis of the music signal and the internal coupling analysis of the correlation degree, the high-intensity integration processing of multiple sets of music signals can be realized. The conversion of “signal-data” realizes the digital processing of music signals.

The process of PSO-BP neural network analysis and big data analysis of audio signal is shown in Figure 2.

In Figure 2, the working principle of the big data analysis center and the PSO-BP neural network is as follows: firstly, the input music signal is analyzed through the self-correlation degree to complete the digital conversion of “audio signal-digital signal,” and then the digital information is input so that the PSO-BP neural network algorithm processing center realizes the classification of the signal through feature analysis and inputs the part of the signal with the coupling correlation to the big data analysis center, and the big data analysis center then performs the “analysis” System mode, learning system mode, and evaluation system to adaptively decouple these signals related to the coupling degree and output information related to their emotions, such as characteristics, expression methods, and judgment criteria, so as to realize the performance of the music signal (sentiment analysis).

### 3.2. Quantitative Evaluation Process of Music Emotion Analysis Model Based on PSO-BP Neural Network

In order to further study the influence of audio signal on music emotion expression under PSO-BP neural network, this study evaluates the simulation results of influencing factors of human music emotion expression through PSO-BP neural network algorithm. This method is a multicriteria decision analysis method which combines qualitative and quantitative analysis. It is the most widely used method for decision analysis of all kinds of problems. It decomposes the relevant factors of decision problems into multiple levels and then makes quantitative analysis. In the analytic hierarchy process (AHP) based on PSO-BP neural network algorithm, the evaluation process is mainly divided into the following steps.

In the first step, the analytic hierarchy process (AHP) system is established. Combined with the research theory of music emotion expression and time-domain signal analysis, the unified analysis is carried out in the process of detecting the change of the simulation signal of music emotion expression. Combined with the PSO-BP neural network audio signal simulation system based on fish swarm recursion theory, the feature extraction algorithm is applied to the simulation model of PSO-BP neural network. Based on the feature extraction algorithm, the PSO-BP neural network music emotion analysis method is established, which is divided into data acquisition, data processing, result feedback, and other parts.

The second step is to determine each index according to different angles and then divide the system into different levels. For the convenience of calculation, the block diagram is often used to illustrate, as shown in Figure 3.

The third step is to determine the maximum eigenvalue of the eigenmatrix in the model *λ*. After normalization, the relative importance ranking is reflected. Although this structure can reduce the interference of other factors and objectively reflect the difference of influence, it is bound to have a certain degree of nonheterogeneity in the comprehensive comparison. If the results are consistent, the discriminant function *a*(*x*) should satisfy the following requirements:

(4) $$\begin{array}{c} a\left(x\right)=\frac{kw\left(x\right)+iw\left(x\right)}{i+k}, \end{array}$$

where *k* and *i* are matrix factors. The process of judging whether the model has passed the consistency test and met the requirements of the consistency test can be recognized as the effective value, as shown in Figure 4.

The fourth step is to check the consistency. At present, the main scaling method is 9-scale method, and its test function QR(*x*) expression is as follows:

(5) $$\begin{array}{c} \text{QR}\left(x\right)=\frac{x^{3}+x^{2}+x+2}{x^{2}+1+x^{-1}}. \end{array}$$

After the index is divided and registered, the value is assigned, the matrix is established, and then the useful information is extracted from the matrix. By constructing pairwise judgment matrix and matrix mathematical method, the importance is ranked. From the perspective of timbre emotionality, too many grades will affect the difficulty of judgment, so the 1–9 scale method is the most reasonable. According to the calculated simulation value to find the corresponding reference value, Table 2 is the average random consistency reference index QR value.

Therefore, in order to reduce the computational complexity of the PSO-BP algorithm, the setting of some parameters in this study is not all obtained by adaptive analysis and training according to the PSO criterion, but a part of the data is directly used by QR reference values. The other part of the threshold setting is obtained by adaptive analysis and deep learning based on a large number of data samples. In this way, it cannot only ensure the accuracy of the PSO-BP neural network algorithm, but also, to a certain extent, reduce the computational complexity of the PSO-BP neural network algorithm and achieve a balance between the accuracy of the solution and the computational complexity.

Finally, the above PSO-BP neural network algorithm and music intervention conditions need to be improved. In this paper, the scaling method is mainly improved, and the 3-scale method is adopted. This method is much simpler to operate. Only through pairwise comparative analysis is the calculation carried out according to the example of importance. If the factors are equally important, 1 shall be used; otherwise 0.5 shall be used. This algorithm also has other defects, such as the tonal rules of music and the simulation process will directly affect the establishment of the judgment matrix. Affected by subjective factors, it is very easy to make objective errors and fail to pass the consistency test. Moreover, these factors are very complex, so it can be verified by simulation. It is found that this method can promote the improvement of timbre quality and the continuous growth of different emotions in the process of national music teaching. Therefore, the analytic hierarchy process cannot objectively reflect the research problems. It also needs to use the fuzzy AHP based on PSO-BP neural network algorithm for evaluation. The evaluation process is shown in Figure 5.

In the process of analyzing the influence factors of PSO-BP neural network on college students' group music emotional expression, the empirical value estimation method is used to determine the fuzzy weight vector, and the membership degree of UU to the coupling value is used for the empirical evaluation. Then the average value of different audio signal group evaluation results is calculated and normalized. In the application of PSO-BP neural network algorithm, it is on the basis of fuzzy evaluation to determine the set of influence degree of national music on music emotional expression under different time length of PSO-BP neural network and then divide the grades to determine the weight value of different influencing factors, so as to realize the quantitative and unified evaluation of the influencing factors of music emotional expression by PSO-BP neural network.

### 3.3. Systematic Design of College Students' Music Emotion Expression Model

Under the intervention of multiple quantitative coupling factors, in order to study the influence of different audio signals on the emotional expression model of music, the accuracy of the simulation is quantitatively analyzed, but in many cases there is no quantitative data, so it is necessary to use the qualitative data in the simulation process (perform quantitative conversion). The method used is to unify the evaluation function. If there is a certain evaluation point in a sequence, and the points can be connected, a unified evaluation function can be generated based on the meeting function. The simulation results show that the interactive model can effectively reduce the influence errors of different PSO-BP neural networks on timbre, can improve the accuracy evaluation of music emotion expression factors and the efficiency of collaboration, and is suitable for different PSO-BP neural networks. In the process of PSO-BP neural network simulation, it can also adapt to subjective interference signals.

In the evaluation of the influence of the PSO-BP neural network on human music emotion expression, the meaning of the data is different, so it is not equal to analysis. The original data needs to be processed in dimensionless mannner, and the linear method is used in this study. After normalization, the relationship of simulation sequences of PSO-BP neural network with different time lengths can be calculated, and then the difference between each factor and the main factor at the same observation point can be calculated. The simulation results are shown in Figure 6.

It can be seen from Figure 6 that the stability of the simulation results of the music emotion analysis model based on PSO-BP is better, and its change law is better than the filtering of the results obtained by the other two methods. In the comprehensive evaluation of the simulation results of the influence of the PSO-BP neural network on college students' music emotion expression, the sequencing problem is involved in most cases. Each evaluation object needs to be sorted first, so it needs to be further compared with the help of gray comprehensive evaluation index.

In order to study the rules of music emotion expression based on PSO-BP neural network and big data analysis, the hierarchical relationship of the gray evaluation index used in this paper is expressed by set, and its expression UU is as follows:

(6) $$\begin{array}{c} {\left\|U_{im}\right\|}_{2}^{2}={\left\|\frac{\sqrt{i^{2}+m^{2}}}{i+m}*\frac{\left(U_{i1},\ldots ,U_{im}\right)}{m}\right\|}_{2}^{2}. \end{array}$$

In the formula, *i* is the sequence number of the signal, and *m* is the disturbance factor.

In the evaluation function of music emotion expression, each secondary indicator will also be expressed by different coefficients. The weight vector function is expressed as *f*(*x*), and its expression is

(7) $$\begin{array}{c} f\left(x\right)=\frac{5x^{3}+2\sqrt{x^{2}+x+2}}{3\sqrt{x^{2}+1+x}}, \end{array}$$

where *x* is the audio signal.

## 4. Result Analysis and Discussion

### 4.1. Evaluation Index of Music Emotion Analysis Experiment Based on PSO-BP Neural Network

In this study, we use five classification methods to evaluate the influence factors of music emotion expression under different neuron nodes. After determining the grading, these grades are assigned a score. Five grades are assigned a five-point method: significantly affects the grading interval [4.5, 5], generally affects the grading interval [3.5, 4.5], basically affects the grading interval [3, 3.5], has little influence on the grading interval [2.5, 3.0], and has no influence on the grading interval [0, 2.5]. The evaluation system of each column is shown in Table 3.

### 4.2. Experimental Results and Analysis

Table 4 is the experimental results of three groups of music emotion analysis under the optimization of PSO-BP neural network. The relevant data in this evaluation model are processed by MATLAB software.

In this research, different types of evaluation criteria are used to achieve quantitative evaluation and characterization, such as combining the popular intelligent evaluation criteria and grouping and characterizing different types of music data, and the evaluation criteria of different data methods are refined (characterization), and then the evaluation result is obtained according to the intelligent data characterization method, and finally a preliminary evaluation and a second evaluation are performed according to the known industry reference standards. In this way, the evaluation and analysis of the experimental results can be completed well, and it is consistent with the current mainstream evaluation rules, and it is more convincing. In order to facilitate the calculation, the various indicators are numbered first, and then the weights are calculated. The experimental analysis results are shown in Figure 7.

As can be seen from Figure 7, the results of PSO-BP neural network model are more stable with the increase of analysis times and are better than the experimental analysis results of several other methods, which shows that, compared with the traditional neural network music analysis model and its optimization algorithm, the music emotion analysis model based on PSO-BP neural network and big data analysis has better analysis effect in the emotion analysis of local music signals. In addition, according to the experimental data and results, the index can be obtained. Finally, the gray comprehensive evaluation value of music emotion expression of different experimental groups is calculated to be 4.0602.

## 5. Conclusion

The current music works have problems such as poor quantification and large errors in the expression of music emotion. Based on this, this paper studies a music emotion analysis model based on PSO-BP neural network and big data analysis. First, it summarizes the current situation of music sentiment analysis and proposes ideas for improvement and optimization based on its existing problems; secondly, it extracts features and formulates classification strategies for different types of music in terms of expressing emotions; secondly, the influencing factors of music emotion expression are comprehensively analyzed using a multidimensional data model, and the related influencing factors are studied, and their influence rules and weight ranking in the process of emotional expression are summarized; finally, experiments are conducted to verify the music sentiment analysis model of this research. The results show that, compared with the conventional method and unoptimized neural network algorithm or BP neural network algorithm, the applied sentiment analysis model proposed by this research has better reliability performance and lower error rate. This is because the PSO-BP neural network algorithm combines the descent adjustment of the weights of the BP standard, through the correction analysis of the network weights and thresholds according to the idea of particle swarm algorithm, to realize the data training and deep learning in the BP neural network, so it is processing. Before data, the data can be roughly searched on a global scale to obtain an initial solution, which reduces the difficulty of subsequent BP neural network analysis, thereby improving the efficiency and accuracy of data analysis. This is also the process of processing music signals in this research, where the innovation is in. However, this study only considered the processing of the simulated signal and did not consider the elimination of other interference signals, so a more in-depth study can be carried out.

## Figures and Tables

**Figure 1:** PSO-BP neural network algorithm processing process of music signal.

**Figure 2:** The process of PSO-BP neural network and big data analysis of audio signals.

**Figure 3:** Analyze the process of each indicator according to different dimensions.

**Figure 4:** The process of model consistency verification.

**Figure 5:** Fuzzy analytic hierarchy process evaluation based on PSO-BP neural network algorithm.

**Figure 6:** Difference between simulated value and reference value.

**Figure 7:** Image after simulation using conventional simulated annealing algorithm.

**Table 1:** Common reference indicators in music sentiment analysis.

Reference indicator type	Reference
Number of voice types	0–90
Number of key audio	0–60
Number of treble and bass types	0–30
Number of mixed audio	0–15

**Table 2:** QR value of average random consistency index.

*n*	1	2	3	4	5	6	7	8	9
QR	0	0.29	0.38	0.51	0.65	0.77	0.86	0.95	1.02

**Table 3:** Sample matrix.

Index	1	2	…	*P*
*U*_11_	*d*_111_	*d*_112_	…	*d*_11*p*_
*U*_12_	*d*_121_	*d*_122_	…	*d*_12*p*_
…	…	…	…	…
*U*_*mn*_	*d*_*mn*1_	*d*_*mn*2_	…	*d*_*mnp*_

**Table 4:** Experimental results of sentiment analysis on 4 sets of music data.

Index	First calculation (4.5)	Second calculation (4.5)	First calculation (5)	Second calculation (5)	Average evaluation value
Experimental group 1	*f*_1_(4.5)	*f*_1_(4.5)	*f*_1_(5)	*f*_1_(5)	0.89
Experimental group 2	*f*_3_(4.5)	*f*_3_(4.5)	*f*_3_(5)	*f*_3_(5)	0.86
Experimental group 3	*f*_4_(4.5)	*f*_4_(4.5)	*f*_4_(5)	*f*_4_(5)	0.99

## Data Availability

The data used to support the findings of this study are available from the corresponding author upon request.
